# Aquaporin 4 Depolarization-Enhanced Transferrin Infiltration Leads to Neuronal Ferroptosis after Subarachnoid Hemorrhage in Mice

**DOI:** 10.1155/2022/8808677

**Published:** 2022-06-17

**Authors:** Yuan Liu, Zongqi Wang, Chang Cao, Zhongmou Xu, Jinxin Lu, Haitao Shen, Xiang Li, Haiying Li, Jiang Wu, Gang Chen

**Affiliations:** ^1^Department of Neurosurgery & Brain and Nerve Research Laboratory, The First Affiliated Hospital of Soochow University, 188 Shizi Street Suzhou Jiangsu Province 215006, China; ^2^Institute of Stroke Research, Soochow University, China

## Abstract

The infiltration of blood components into the brain parenchyma through the lymphoid system is an important cause of subarachnoid hemorrhage injury. AQP4, a water channel protein located at the astrocyte foot, has been reported to regulate blood–brain barrier integrity, and its polarization is disrupted after SAH. Neuronal ferroptosis is involved in subarachnoid hemorrhage- (SAH-) induced brain injury, but the inducing factors are not completely clear. Transferrin is one of the inducing factors of ferroptosis. This study is aimed at researching the role and mechanism of AQP4 in brain injury after subarachnoid hemorrhage in mice. An experimental mouse SAH model was established by endovascular perforation. An AAV vector encoding AQP4 with a GFAP-specific promoter was administered to mice to achieve specific overexpression of AQP4 in astrocytes. PI staining, Fer-1 intervention, and transmission electron microscopy were used to detect neuronal ferroptosis, and dextran (40 kD) leakage was used to detect BBB integrity. Western blot analysis of perfused brain tissue protein samples was used to detect transferrin infiltration. First, neuronal ferroptosis 24 h after SAH was observed by PI staining and Fer-1 intervention. Second, a significant increase in transferrin infiltration was found in the brain parenchyma 24 h after SAH modeling, while transferrin content was positively correlated with neuronal ferroptosis. Then, we observed that AQP4 overexpression effectively improved AQP depolarization and BBB injury induced by SAH and significantly reduced transferrin infiltration and neuronal ferroptosis after SAH. Finally, we found that AQP4 overexpression could effectively improve the neurobehavioral ability of SAH mice, and the neurobehavioral ability was negatively correlated with transferrin brain content. Taken together, these data indicate that overexpression of AQP4 in the mouse brain can effectively improve post-SAH neuronal ferroptosis and brain injury, at least partly by inhibiting transferrin infiltration into the brain parenchyma in the glymphatic system.

## 1. Introduction

Stroke is divided into ischemic stroke and hemorrhagic stroke, and hemorrhagic stroke accounts for 20%~30% of all strokes [1]. Although the incidence of hemorrhagic stroke is lower than that of ischemic stroke, its prognosis is worse, and its mortality and disability rates are higher than those of ischemic stroke [2]. Subarachnoid hemorrhage caused by ruptured intracranial aneurysm is one of the main forms of hemorrhagic stroke, with an annual incidence of approximately 10.5/100,000 people in China [3]. At present, there have been a large number of experimental studies on the intervention of brain injury after stroke, but the results of experimental studies have little effect in clinical application [4]. The scientific prevention and treatment of brain injury after SAH is an urgent problem in today's society [1].

Neuronal death is an important component of brain injury after SAH [5]. An increasing number of studies suggest that SAH triggers neuronal ferroptosis [6–8], and intervention with ferroptosis inhibitors is beneficial for improving early brain injury (EBI) after SAH [9, 10]. Mature neurons have a high level of polyunsaturated ether phospholipids (PUFA-EPLS), which makes them sensitive to ferroptosis [11, 12]. Glutamine (0.1 mm) and recombinant transferrin (0.25-5 *μ*g/mL) caused ferroptosis in mouse embryonic fibroblasts (MEFs) deprived of amino acids [13]. The normal medium of primary cortical neurons contained 0.5-2 mM glutamine, suggesting that the environment of neurons was rich in glutamine. Transferrin is not typically expressed by neurons, but it is absorbed by neurons through TFR1-mediated endocytosis, which is the primary source of iron in neurons [14]. Blood is known to be rich in transferrin [15]. Therefore, it is worth considering whether transferrin enters the glymphoid system after SAH infiltrates the brain parenchyma and participates in neuronal ferroptosis.

The glymphoid system is a channel for the exchange of cerebrovascular cerebrospinal fluid and interstitial fluid, distributed in the Virchow-Robin space and perivascular space (PVS) [16]. Privious research has stated “Bathing the brain” to describe the role of the glymphoid system under physiological conditions [17]. PVS includes the spaces around small cerebral arteries, capillaries, and venules, which constitute channels that allow a range of substances to move [18]. Within a few minutes of the occurrence of SAH, blood components rapidly diffuse into the subarachnoid space and PVS [19]. Loss of astrocyte foot process anchoring to the basement membrane accompanied by the loss of polarized localization of AQP4 to astrocytic endfeet has been shown to be associated with vasogenic/extracellular edema in neuroinflammation [20]. In addition, it has been shown that SAH impairs the polarization of astrocyte AQP4 [21], while AQP4 knockout aggravates SAH-induced brain injury through impairment of the glymphoid system [22]. In addition, literature studies have shown that upregulation of AQP4 improves blood–brain barrier integrity and perihematomal edema following intracerebral hemorrhage [23].

Here, we investigated the occurrence and possible initiator of neuronal ferroptosis after SAH in mice. By using propidium iodide (PI) staining, we provided a description of the correlation between brain cell ferroptosis and transferrin content, alluding to the critical role of transferrin in SAH-induced brain cell ferroptosis. We assessed the effect of AQP4 overexpression on transferrin content as well as brain cell ferroptosis. Finally, we demonstrated that AQP4 overexpression effectively improved the neurobehavioral ability of SAH mice. In this study, we provide the first demonstration of transferrin function in an animal model of SAH and establish the essential role of AQP4 in regulating transferrin infiltration into the brain parenchyma.

## 2. Materials and Methods

### 2.1. Animals

Five to 8-week-old C57BL/6J male mice weighing 25-30 g were purchased from Zhaoyan Research Center (Suzhou, China) Co., Ltd. Standard feed and drinking water were provided. This study was approved by the Ethics Committee of the First Affiliated Hospital of Soochow University. Detailed animal usage information is provided in the supplementary material 1 (Supplementary Table S1).

### 2.2. Mouse SAH Model

The endovascular perforation method was used to establish the mouse SAH model as previously reported [24, 25]. Mice were anesthetized with 3% isoflurane using a small animal gas anesthesia machine (R500IP; RWD Life Technology Co., Shenzhen, China), and anesthesia was maintained with 1.5% isoflurane [26]. Then, they were placed in a stereotaxic apparatus (Anhui Zhenghua Biological Equipment Co., Ltd., Anhui, China). The mice were placed in a supine position, and a midline incision was made in the neck. After exposing the right common carotid artery (CCA), external carotid artery (ECA), and internal carotid artery ICA, the ECA was ligated and fashioned into a stump. The suture (L2000, Guangzhou Jialing) was advanced into the ICA from the ECA stump through the common carotid bifurcation. The suture was further advanced into the intracranial ICA until resistance was felt. Before the suture was withdrawn from the ICA, it was pushed an additional 1 mm further. After ensuring hemostasis, the wound was adapted and sutured. For the sham-operated animals, all procedures were the same as those for the SAH mice, except for artery puncture. Then, all the mice were returned to their cages after injecting 1 ml 0.9% saline. All mice had free access to food and water. The grade of SAH was evaluated with a score of 0-18 to measure the degree of bleeding and was carried out by two researchers who were unaware of the experiment. Images of the bottom of the brain were taken, and the 6 segments at the bottom of the basal cistern were evaluated on a scale from 0 to 3 (0, no SAH; 1, very little subarachnoid blood; 2, moderate blood with visible arteries; and 3, blood clot obliterating all arteries within the segment). Finally, the scores of each part are summed. Mice with SAH classification scores < 8 were excluded and replaced. In sham-operated mice, the score is always 0.

### 2.3. Ferrostatin-1 Treatment

For in vivo experiments, we injected 1 pmol ferrostatin-1 (1 *μ*l of 25 mg Fer-1 dissolved in 0.01% DMSO saline, Sigma Aldrich, SML0583) into the lateral ventricle immediately after 0.5 h of SAH modeling and simultaneously injected 1 *μ*l solvent into the control group in the same way [27]. The coordinates of intraventricular injection were 1.0 mm in the lateral direction relative to the bregma, 0.5 mm in the posterior direction, and 2.5 mm in depth. After 24 hours, the head was decapitated, and the brain tissue was harvested. PI dye (Sigma–Aldrich, St. Louis, MO, USA) (1 *μ*g/g) was injected intraperitoneally 2 hours before the head was decapitated.

### 2.4. Immunofluorescence Staining

As previously reported, brain tissue was cut into 7 *μ*m paraffin sections [28]. Briefly, the antigens were retrieved using freshly prepared 1% sodium citrate antigen retrieval solution for 20 min. The paraffin sections were boiled in antigen retrieval solution for 5 min and then soaked in cooled antigen retrieval solution for 5 min. The above operation was repeated twice. Next, 0.1% Triton was added for 10 min. After that, we used 5% BSA to block these sections for 1 h at room temperature. The target protein primary antibody was added according to the manual, and the solution was incubated overnight at 4°C. The primary antibodies were as follows: AQP4 rabbit mAb (1 : 300, Cell Signaling Technology, #59678, USA) and goat CD31 antibody (1 : 300, R&D systems, AF3628, USA). Then, the corresponding fluorescent secondary antibody was added. The secondary antibodies were as follows: donkey anti-rabbit IgG Alexa Fluor 488 (1 : 300, Thermo Fisher Scientific, A-21206, USA) and donkey anti-goat IgG Alexa Fluor 555 (Thermo Fisher Scientific, A-21432, USA). The solution was incubated at 37°C for 1.5 h [26]. Brain sections were sealed with DAPI and observed under a fluorescence microscope. Coronal brain sections containing the basal temporal lobe were analyzed (Fig. S2).

### 2.5. Propidium Iodide (PI) Staining

As previously reported, twenty-two hours after the establishment of the SAH model, mice were injected with PI (Sigma–Aldrich, St. Louis, MO, USA) (1 *μ*g/g) intraperitoneally [29]. After 2 hours, they were perfused with PBS, the heads were decapitated, and the materials were removed. After being fixed with paraformaldehyde for 24 hours, they were dehydrated with 30% sucrose. Then, brain tissue was cut into 8 *μ*m sections in the dark and under freezing conditions. Quick Antigen Retrieval Solution for Frozen Sections (Beyotime, P0090) was added for 10 min. Next, 0.1% Triton was added for 10 min, and 5% BSA was used to block these sections for 1 h at room temperature. The target protein primary antibody was added, and the solution was incubated overnight at 4°C. The primary antibody was mouse anti-NeuN (1 : 300, Abcam, ab279296, USA). Then, the corresponding fluorescent secondary antibody was added, and the solution was incubated at 37°C for 1.5 h. The secondary antibodies were as follows: donkey anti-mouse IgG Alexa Fluor 488 (1 : 300, Thermo Fisher Scientific, A-21202, USA). Brain sections were sealed with DAPI and observed under a fluorescence microscope (OLYMPUS BX50/BX-FLA/DP70; Olympus Co.). Coronal brain sections containing the basal temporal lobe were analyzed (Fig. S2). In short, PI+/NeuN+ cells were counted by observers who were blinded to the experimental groups. We inspected and photographed six microscopic fields of each sample and calculated the average.

### 2.6. Western Blot Analysis

The brain tissues were collected from the base of the temporal lobe and stored immediately at −80°C. As previously reported, the temporal base brain tissues of C57 mice were collected and homogenized in cell lysate buffer for Western blotting and IP (P0013, Beyotime Institute of Biotechnology, China) and allowed to stand for 30 minutes. The tissue homogenate was collected into a centrifuge tube and centrifuged at 12,000 rpm/min for 10 minutes at 4°C. The supernatant was taken, and the protein concentration was measured by the bicinchoninic acid assay (BCA, Beyotime Institute of Biotechnology) [30]. Then, each protein sample (10~60 *μ*g/lane) was loaded on a 10% SDS–PAGE gel, separated by electrophoresis, and transferred to a polyvinylidene fluoride membrane by electrophoresis (Millipore Corporation, Billerica, MA, USA), followed by blocking with 5% BSA at room temperature for 60 minutes and then incubating with primary antibody overnight at 4°C. The primary antibodies were as follows: rabbit anti-transferrin antibody (1 : 1000, Abcam, ab278498, USA) and *β*-tubulin (9F3) rabbit mAb (1 : 1000, Cell Signaling Technology, #2128, USA). The diluted horseradish peroxidase-labeled secondary antibody was incubated at room temperature for approximately 1 hour and then washed with PBST (PBS+0.05% Tween 20) 3 times for 5 minutes each. The secondary antibodies were as follows: anti-rabbit IgG and HRP-linked antibody (1 : 2000, Cell Signaling Technology, #7074, USA). After the Ponceau was stained and washed off, the enhanced chemiluminescence kit was used for band visualization, and then, the protein relative quantitative normalization analysis was performed by the ImageJ software. Detailed antibody information is provided in the supplementary material 1 (Supplementary Tables S3, S4 and S5). Full Western blot lane is presented in supplementary material 2.

### 2.7. Stereotaxic Adenoassociated Virus Injection

AAV9-AQP4 containing adenoassociated virus GFAP-MCS-EGFP was used for overexpression of AQP4 protein (NM_009700.3→NP_033830.2 aquaporin-4 isoform M1) in mouse astrocytes and its negative control (Jike gene; GenBank: NM-009700) and stored at -80°C. According to the manufacturer's instructions, 1 *μ*l adenoassociated virus (1.1*E* + 13 v.g/ml) was injected into the lateral ventricle. The coordinates from bregma were 1.0 mm posterior, 1.8 mm lateral, and 2.4 mm deep [21]. Leave the needle for 5 minutes after the AAV injection and then pull it out slowly. We established an SAH model three weeks after AAV9-AQP4 injection. Detailed AAV information is provided in the supplementary material 1 (Supplementary Table S2).

### 2.8. Quantification of AQP4 Polarization

Perivascular polarization of AQP4 was measured as previously described [31]. DAPI images were used to identify blood vessels. Blood vessels have flattened nuclei and clusters or lines of nuclei out of focus compared to the surrounding tissue. CD31 images were used to identify the astrocytes around the blood vessels [32]. Briefly, the median immunofluorescence intensity of perivascular regions was measured. A threshold analysis was then used to measure the percentage of the region exhibiting AQP4 immunofluorescence greater than or equal to perivascular AQP4 immunofluorescence (AQP4% area). Polarization was expressed as the percentage of the region that exhibited lower AQP4 immunoreactivity than the perivascular endfeet (^“^polarization^”^ = 100–AQP4%area). AQP4 vessel coverage was measured by first delineating the area of the vessel from the CD31 channel image. This region of interest was then placed on the AQP4 channel image thresholded for immunoreactivity for extraction of the percentage vessel coverage (% immunoreactivity of AQP4 of whole delineated vessel).

### 2.9. FITC-Dextran (40 kD) Injection

Briefly, FITC-dextran (40 kD, Thermo Fisher, D3328) was injected intravenously 21 hours post-SAH [33]. The mice were sacrificed 3 hours following tracer infusions, perfused, and fixed with paraformaldehyde. Brains were removed and cut into 10 *μ*m slices. Cerebrovascular permeability was evaluated by fluorescence imaging.

### 2.10. Electron Microscopy

Briefly, the brain tissue sections were postfixed with 4% paraformaldehyde +2.5% glutaraldehyde in 0.1 M PB for 14 hours at 4°C. Then, they were washed and stored in 0.1 M PB [34]. The coverslips were processed for electron microscopy as previously described with modifications [35]. Ultrathin sections at 70-80 nm were cut on an ultramicrotome and collected on Formvar-coated single slot grids (Electron Microscopy Sciences). Grids were stained with uranyl acetate and lead citrate solutions, dried, and stored in a grid box for EM imaging. Micrographs were taken on a Tecnai Biotwin transmission electron microscope (FEI, Hillsboro, Oregon, USA). We measured mitochondrial size as the percentage area of the total area of the cytoplasm [36] (comprising >1800 mitochondria in total) using ImageJ v.1.49 (http://imagej.nih.gov/ij/). Analysis was performed by an investigator blinded to treatment group assignment.

### 2.11. Foot Fault Test

As previously reported, the mouse was placed on an elevated steel grid (30 cm (*L*) × 35 cm (*W*) × 3 cm (*H*)) with a grid opening of 2.25 cm 2 (1.5 cm × 1.5 cm square) [37, 38]. The mice received 5 days of pretraining before the operation. The data in the last training session were recorded as baseline. The total number of steps was counted for a videotaped 1-minute observation period. The number of forelimb and posterior limb foot faults (when the forelimb or posterior limb fell through the grid) was recorded. The data were collected by unwitting staff. The data are expressed as the percentage of errors with damage to the forelimb and posterior limb. This test will be repeated three times at the indicated times after the operation, recorded separately, and averaged.

### 2.12. Adhesive Removal Test

As previously reported, the sticker (0.2 × 0.2 cm^2^) was placed on the paw on the inner radius of each animal's upper limb with equal pressure [37]. The stickers were placed on the left forelimbs of each animal. Then, the mouse was gently placed into the plexiglass box, and the number of seconds to touch and remove each tape was recorded. The mice were trained 3 times a day before surgery for 5 consecutive days and were tested regularly (3 times, 15 minutes apart for each mouse) at the indicated times after SAH [26]. The average time of the three trials of touching and removing the sticker will be calculated.

### 2.13. Rotarod Test

As previously reported, low speed: the instrument is set to accelerate from 0 rpm to 10 rpm within 30 s and maintained to 300 s; high speed: the instrument is set to accelerate from 4 rpm to 40 rpm and maintained to 300 s within 120 s [39, 40]. The mice will be placed on a rotating rod apparatus, and preoperative training will continue for 5 days. On the first and second days, the mice will be trained on a low-speed rotating rod once a day. On the third day, low-speed and high-speed training will be carried out successively. Then, on the fourth day, the mice were trained twice at high speed at the test speed. High-speed training was performed three times on the fifth day. The last three test data recorded the day before the operation were taken as the baseline. The mice were subjected to three tests at the indicated times after the SAH operation, with an interval of 15 minutes, and the average value was taken [26].

### 2.14. Garcia Neuroscore

The sensorimotor Garcia test was performed on mice at the indicated times after SAH [41]. In short, the modified Garcia score is a complete sensorimotor evaluation system. We scored each test from 0 to 3 (full score = 18 points): (A) body proprioception, (B) forelimb walking, (C) limb symmetry, (D) roll over, and (E) climb. Autonomous movement: in a quiet environment, place the mouse in a new squirrel cage, observe its activity within 5 minutes, and score according to the number of touches on the four sides of the cage wall; autonomous movement of the limbs: move the mouse and lift the tail end to observe the free movement and symmetry of its limbs; forelimb extension exercise: lift the tail end of the mouse so that its forelimbs are close to the edge of the table, and observe the extension of its forelimbs; metal net climbing: place the mouse on the tilted metal cage cover and observe its climbing situation. Normal mice will climb up with their limbs. Lift the tail of the mouse and drag it away from the cage cover to observe the grasping power of its limbs; body tactile response: in a quiet environment, from back to front, avoiding the sight of the mouse, touch the body of the mouse with a blunt-headed wooden stick to observe its response; whisker response: in a quiet environment, use a blunt-headed wooden stick to touch the rat from the back side; response to vibrissae touch: in a quiet environment, a blunt stick was brushed against the vibrissae on each side; the stick was moved toward the whiskers from the rear of the animal to avoid entering the visual fields. The reaction of mice was observed.

### 2.15. qPCR

The mRNA expression of AQP4 (NM_009700.3) was measured as previously described [42]. Briefly, total RNA was isolated from the brain tissues of mice using the TRIzol kit (15596018, Thermo Fisher, US) and reverse transcribed into cDNA (2 *μ*g total RNA per sample) using the High-Capacity cDNA Reverse Transcription Kit (4368814, Thermo Fisher, USA) according to the manufacturer's instructions. The primer sequences used for the reaction were AGATCAGCATCGCTAAGTCCGT TCCCAATCCTCCAACCACAC (Ribobio, China). qPCR was performed using the PowerUp™ SYBR™ Green Master Mix, and mRNA expression levels were quantified using the 2^−∆∆Ct^ method.

### 2.16. Statistical Analysis

All data are expressed as the mean ± standard deviation (SD). The GraphPad Prism 9.0 software (GraphPad, San Diego, CA, USA) was used for statistical analysis. Post hoc power analysis was performed according to power analysis. The Kolmogorov–Smirnov test was used to test the normality of the distribution of the test data set. Data groups with normal distribution (two groups) were compared using two-sided unpaired Student's *t*-test. One-way or two-way ANOVA was used for multiple comparisons, and Tukey's post hoc test was used for comparisons between two pairs of multiple groups. *P* < 0.05 indicates a statistically significant difference. The correlation between transferrin and PI staining was analyzed with Spearman's rank correlation coefficient for the neuroscore and beam walking score. For the Garcia neuroscore, adhesive removal, foot fault tests, and rotarod test, the correlation between neurobehavior and transferrin was analyzed with Pearson's product–moment correlation coefficient. The best-fit linear regressions are shown. A *P* value of 0.05 was considered statistically significant.

## 3. Results

### 3.1. SAH Triggers Brain Cell Ferroptosis and Transferrin Infiltration

Ferrostatin-1 is a recognized ferroptosis inhibitor [27]. To verify the existence of ferroptosis of nerve cells after SAH in mice, we used Fer-1 intraventricular injection after surgery. The results showed that compared with the vehicle group, the Fer-1 group had significantly reduced neuronal death (sham vs. SAH, *P* < 0.0001; SAH vs. SAH+vehicle, *P* = 0.9888; and SAH+vehicle vs. SAH+Fer-1, *P* = 0.0119; Figures 1(a) and 1(b)). This phenomenon indicates ferroptosis in mouse brain cells after SAH. Transferrin is an important factor in ferroptosis in cells [13]. Twenty-four hours after puncture-induced SAH in mice, brain tissues from the base of the temporal lobe were collected for western blot analysis. Our results showed that compared with that in the sham group, the expression of transferrin in the SAH group was increased (sham vs. SAH, *P* = 0.0002; Figure 1(c)). Next, we measured the correlation between the expression of transferrin and PI+ nerve cells. The results showed that there was a significant positive correlation between the number of PI+ cells and the expression of transferrin (Figure 1(d)). The above results show that SAH triggers brain cell ferroptosis and transferrin infiltration.

### 3.2. AQP4 Overexpression Improves SAH-Induced AQP4 Depolarization

qPCR was used to detect the expression level of AQP4 mRNA in brain tissue after AAV-AQP4 overexpression. Our results showed that the expression level of AQP4 mRNA in the AAV-AQP4 group was approximately 2-fold that in the vector group (*P* = 0.0427, Fig. S1). To further explore this possibility, we assessed the level of AQP4 using immunofluorescence staining. Twenty-four hours after SAH, the AQP4 level in astrocytes was significantly decreased compared with that in the sham group, and compared with that in the SAH+vector group, AAV-AQP4 significantly increased the expression of AQP4 (sham vs. SAH, *P* < 0.0001; SAH vs. SAH+vector, *P* = 0.9945; and SAH+vector vs. SAH+AAV-AQP4, *P* < 0.0001; Figures 2(a), 2(g), and 2(e)). Vascular cross-sectional analysis of the temporal cortex from mice revealed impaired perivascular AQP4 expression after SAH (Figures 2(b), 2(c), 2(h), and 2(i)). Perivascular localization of AQP4 was reduced, and polarization was reduced. SAH+AAV-AQP4 reversed this change compared to the SAH+vector group. 89.01% (±2.74%), 72.34% (±2.90%), 72.90% (±2.11%), and 80.23% (±2.32%) are in the cortex of mice (sham vs. SAH, *P* < 0.0001; SAH vs. SAH+vector, *P* = 0.9809; and SAH+vector vs. SAH+AAV-AQP4, *P* = 0.0004; Figure 2(g)). Together, these data provide evidence that astrocytic AQP4 expression and its polarized localization are similarly perturbed in a region of the SAH mouse brain.

### 3.3. AQP4 Overexpression Reduces Transferrin Content and Neuronal Ferroptosis in the Brain Parenchyma of SAH Mice

The effects of AAV-AQP4 on BBB integrity in SAH model mice were assessed by a FITC-dextran permeability assay [33]. At 24 h after SAH, 40 kD dextran extravasation was detected in the mouse brain parenchyma, which was improved to some extent by AAV-AQP4 treatment (Figure 3(a)). We evaluated the expression of transferrin using Western blotting. Compared with the vector treatment group, the transferrin expression level in the AQP4 overexpression group was significantly decreased (SAH vs. SAH+vector, *P* = 0.9146 and SAH+vector vs. SAH+AAV-AQP4, *P* = 0.0053; Figures 3(b) and 3(c)). We used PI staining to evaluate the death of neurons after SAH. Our results showed that the number of neurons containing PI in the SAH+vector group was significantly higher than that in the SAH+AAV-AQP4 group, and there were no significant changes in the SAH+AAV-AQP4+vehicle group compared with the SAH+AAV-AQP4 group (SAH+vector vs. SAH+AAV-AQP4, *P* < 0.0001 and SAH+AAV-AQP4 vs. SAH+AAV-AQP4+vehicle, *P* = 0.9943; Figures 3(d) and 3(e)). There were no significant changes in the SAH+AAV-AQP4+vehicle group compared with the SAH+AAV-AQP4+Fer-1 group (*P* = 0.9992). The results showed that overexpression of AQP4 reduced ferroptosis in neurons after SAH in mice. In ferroptosis, shrunken mitochondria have been observed, while the formation of apoptotic bodies was absent, and the plasma membrane remained intact [43]. As the sole positive morphologic criterion for ferroptosis is shrunken mitochondria, we quantified mitochondrial size following AAV-AQP4 treatment. AAV-AQP4 treatment increased the mean percentage area of cytoplasm covered by mitochondria (SAH+vector vs. SAH+AAV-AQP4, *P* = 0.0186; Figures 3(f) and 3(g)). These results indicate that overexpression of AQP4 can reduce transferrin and neuronal ferroptosis in brain tissue after SAH.

### 3.4. AQP4 Overexpression Improves Neurobehavioral Dysfunction in SAH Mice

Mice developed sensorimotor impairment after stroke, which was manifested by a decrease in Garcia neuroscore, an increase in the number of foot faults, an increase in the time of the adhesive removal test, and a decrease in the time of the rotarod test (Figures 4(a)–4(f)). To evaluate the neurological damage after SAH in mice, the evaluation was carried out by researchers who did not know the group. The results showed that compared with the baseline, the Garcia score of the mice decreased significantly one, two, three, and seven days after SAH. Compared with the vehicle group, the Garcia score of the AAV-AQP4 group was significantly improved on day 3 (SAH+vector vs. SAH+AAV-AQP4, *P* = 0.0296; Figure 4(a)). Compared with the baseline, the proportion of the number of wrong steps in the contralateral forelimbs and hindlimbs of mice after SAH was significantly increased. AQP4 treatment significantly reduced the percentage of incorrect steps three days after SAH (SAH+vector vs. SAH+AAV-AQP4, day 1, *P* = 0.0079; day 2, *P* = 0.0133; and day 3, *P* = 0.0008; Figure 4(b). SAH+vector vs. SAH+AAV-AQP4, day 1, *P* = 0.0002; day 2, *P* = 0.0207; and day 3, *P* = 0.0038; Figure 4(c)). At the same time, we found that compared with the vehicle treatment group, the waiting time for SAH mice in the AQP4 treatment group to touch and remove the tape from the paw was significantly reduced at 1, 2, 3, and 5 days after SAH (SAH+vector vs. SAH+AAV-AQP4, day 1, *P* = 0.0066; day 2, *P* = 0.0019; day 3, *P* = 0.0004; and day 5, *P* = 0.0002; Figure 4(d). SAH+vector vs. SAH+AAV-AQP4, day 1, *P* = 0.0174; day 2, *P* = 0.002; day 3, *P* = 0.0154; and day 5, *P* = 0.0002; Figure 4(e)). In addition, in the mice in the AQP4 treatment group, on days 1, 2, 3, and 5 after SAH, compared with the vehicle treatment group, the rod time in the rod rotation experiment was slightly increased (SAH+vector vs. SAH+AAV-AQP4, day 1, *P* < 0.0001; day 2, *P* < 0.0001; day 3, *P* < 0.0001; and day 5, *P* = 0.0197; Figure 4(f)). Overall, AQP4 treatment significantly improved the early sensory and dyskinesias of SAH in mice.

### 3.5. Neurobehavioral Ability Was Negatively Correlated with Transferrin Brain Content in SAH Mice

The results of Pearson correlation analysis showed that there was a significant negative correlation between the Garcia score (*R* = −0.8746, *P* < 0.0001), the residence time of the rod (*R* = −0.7088, *P* < 0.0001), and the expression of transferrin after 24 h of SAH (Figures 5(a) and 5(f)). At the same time, there was a significant positive correlation between the foot fault rate (*R* = 0.7481, *R* < 0.0001; *R* = 0.7368, *R* < 0.0001) as well as the adhesive removal test time (*R* = 0.7485, *P* < 0.0001; *R* = 0.7368, *P* < 0.0001) and the expression level of transferrin (Figures 5(b)–5(e)). Overall, neurobehavioral ability was negatively correlated with transferrin brain content in SAH mice.

## 4. Discussion

Ferroptosis has drawn wide attention since the term was put forward in 2012 [43]. This unique cell death program is driven by iron-dependent phospholipid peroxidation and is modulated by multiple cellular metabolic pathways, including redox homeostasis, iron metabolism, and mitochondrial activity [44]. Neuronal death after SAH is an important factor affecting prognosis [45]. Previous studies have shown that neuronal ferroptosis occurs after SAH, but the mechanism is unclear [46]. In addition, neurons have high levels of PUFA-EPLS and live in an environment rich in glutamine, which makes mature neurons sensitive to ferroptosis [12]. Studies have shown that 1 minute after the modeling of the intravascular puncture SAH model in mice, the erythrocyte flow rate and blood flow in the anterior capillary arteriole decreased to 20% of those before modeling [47]. Subsequently, the arterioles dilated or contracted inconsistently for 60 minutes, and the red blood cell flow and blood flow in the arterioles continued to decrease, suggesting neurovascular dysfunction [47]. The results obtained in these studies indicate that the transient disturbance of microcirculation after SAH in the acute phase may lead to oxidative stress, which in turn mediates ferroptosis. Therefore, ferroptosis may play a more important role in brain injury than the current understanding. The focus of this study was to clarify the factors that induce neuronal ferroptosis after SAH and the role of AQP4 in this process.

AQP4 is not just involved in ferroptosis; previous studies have shown that AQP4 knockout aggravates brain edema, blood–brain barrier disruption, and neuronal apoptosis after subarachnoid hemorrhage [22, 48]. Consistent with our study, it has been reported that the perivascular polarity of AQP4 is reduced after SAH in rats, leading to dysfunction of the glymphatic system and neuronal apoptosis and neurological deficits after SAH [21]. In addition, in a mouse model of intracerebral hemorrhage, AQP4 reduction increases neuronal apoptosis and astrocyte apoptosis after intracerebral hemorrhage, and the underlying mechanism may be through cytokines, especially TNF-*α* and IL-1*β* initiate the apoptotic cascade and activate caspase-3 and caspase-8 [49]. In addition, in a rat model of ischemia–reperfusion, induction of pyroptosis leads to loss of AQP4 polarization, which can be ameliorated by inhibition of pyroptosis [50]. The process and mechanism of AQP4 involvement in various forms of programmed cell death deserve further study.

Previous studies have focused on the neurotoxicity of erythrocyte lysis products such as iron, hemoglobin, and heme for neuronal death after SAH [27, 35]. However, less attention has been given to transient microcirculation disorders and the blood component transferrin in the early stages of SAH. Our work suggests that the infiltration of transferrin into the brain parenchyma at the early stage of SAH may be one of the causes of neuronal ferroptosis.

Aquaporin (AQP) is abundant in the brain and spinal cord, and AQP1 and AQP4 are believed to play an important role in water metabolism and osmotic regulation [51]. In the early stage of SAH, blood components rapidly diffuse into the subarachnoid space and the glymphoid system in the PVS [19]. After SAH, microglia/macrophages can remove blood components in the glymphoid system [52]. Enhanced PVS barrier action can make time for blood component clearance [53]. PVS permeability has been reported to have a circadian rhythm and is closely related to AQP4 polarization [20]. It has been reported that the increased expression of AQP4 in rats after subarachnoid hemorrhage will aggravate the occurrence of cerebral edema [54], and the inhibition of AQP4 can inhibit cerebral edema [55, 56]. In addition, studies have shown that the nervous system function of *AQP4^−/−^* mice was improved in a model of cytotoxic edema simulated by intraventricular injection of Streptococcus [57]. However, brain swelling and clinical outcomes are worse in AQP4-/- mice in models of vasogenic (fluid leak) edema, probably due to impaired AQP4-dependent brain water clearance [57]. AQP4 mediates bidirectional water flux as well as water inflow and outflow during the evolution of edema [58, 59]. AQP4 dysfunction in mouse brain tissue leads to impaired water and solute processing and may lead to brain edema or abnormal protein accumulation [60, 61]. Although some studies have shown that AQP4 is involved in brain edema after SAH [62], in recent years, AQP4 knockout has been found to aggravate brain injury after SAH [23], suggesting the functional diversity and potential neuroprotective effect of AQP4. Our work is the first to show that AQP4 overexpression can reduce SAH-induced AQP4 depolarization, brain parenchymal ferritin content, and neuronal ferroptosis to a certain extent.

Stroke affects both men and women, and studies revealed that estrogen has a protective effect after subarachnoid hemorrhage [63]. Our study just used male animals. We will consider gender factors in our subsequent studies to explain the role of AQP4 in animals of different genders after subarachnoid hemorrhage.

In conclusion, in the early stage of SAH, transient disturbance of microcirculation and transferrin induced neuronal oxidative stress and iron uptake, leading to neuronal ferroptosis. Overexpression of AQP4 can improve SAH-induced AQP4 depolarization and transferrin infiltration and thus improve neuronal ferroptosis and neurological dysfunction (Figure 6).

## Figures and Tables

**Figure 1:** SAH triggers brain cell ferroptosis and transferrin infiltration. (a, b) Representative photomicrographs and quantification of PI-positive nerve cells in the ipsilateral cortex after Fer-1 was used. *n* = 6 per group. Fluorescence colors: DAPI: blue; PI: red; NeuN: green. Scale bar = 40 *μ*m. The quantification of PI-positive and NeuN-positive cells is expressed as positive cells per square millimeter. Data are the mean ± standard deviation (SD) (ANOVA *F*(3, 20) = 42.78*P* < 0.0001; ^∗∗∗^*P* < 0.001, ^∗^*P* = 0.0119, post hoc Tukey's test). (c) Western blot analysis shows the level of transferrin protein in the ipsilateral cortex after SAH. *n* = 12 per group. Data are the mean ± standard deviation (SD) (*t*-test *t*_(11)_ = 4.511; ^∗∗∗^*P* < 0.001). (d) Spearman correlation analysis between transferrin- and PI-positive cells in mouse brain tissue 24 h after SAH.

**Figure 2:** AQP4 overexpression improves SAH-induced AQP4 depolarization. (a, g) Immunofluorescence staining analysis of perivascular AQP4 expression changes in mouse temporal cortex large vessels 24 h after SAH. *n* = 6 per group. CD31: red, AQP4: green; DAPI: blue. Scale bar = 20 *μ*m. Data are the mean ± standard deviation (SD). (b, c, h, i) Representative immunofluorescence images of blood vessels in the cortex of (b) sham, (c) SAH, (h) SAH+vector, and (i) SAH+AAV-AQP4 group mice stained for AQP4 and CD31, illustrating placement of the 40 *μ*m axis perpendicular to blood vessels for quantification of expression across vessel cross-sections, illustrating AQP4 expression surrounding blood vessels in the cortex. Ten cross-sections of one blood vessel from one mouse were selected. (d) Viral vector pattern diagram. (e) Immunofluorescence intensity statistics for AQP4. Data are the mean ± standard deviation (SD) (ANOVA *F*(3, 20) = 88.80*P* < 0.0001; ^∗∗∗^*P* < 0.001, post hoc Tukey's test). (f) Quantification of AQP4 polarization. *n* = 6 per group (ANOVA *F*(3, 20) = 56.75*P* < 0.0001; ^∗∗∗^*P* < 0.001; post hoc Tukey's test).

**Figure 3:** AQP4 overexpression reduces transferrin content and neuronal ferroptosis in the brain parenchyma of SAH mice. (a) Representative images of FITC-dextran (40 kD) after post-SAH intravenous injections at 24 hours after SAH (scale bar = 50 *μ*m). (b, c) Western blot analysis showed the levels of transferrin in the cortex after AAV overexpression of AQP4. *n* = 6 per group. Data are the mean ± SD (ANOVA *F*(2, 15) = 8.3*P* = 0.0036; ^∗∗^*P* = 0.0053, post hoc Tukey's test). (d, e) Representative fluorescence micrographs and quantification of PI-positive and neuron-positive cells in the cortex after AAV overexpression of AQP4, *n* = 6 per group. Fluorescence colors: NeuN: green; PI: red; DAPI: blue. Scale bar = 20 *μ*m. The quantification of PI-positive and NeuN-positive neurons is expressed as positive cells per square millimeter. Data are the mean ± SD (ANOVA *F*(3, 20) = 157.2*P* < 0.0001; ^∗∗∗^*P* < 0.001, post hoc Tukey's test). (f) Electron microscopic images of the SAH+vector group and SAH+AAV-AQP4 group. (g) AAV-AQP4 treatment reduced the mean percentage area of cytoplasm covered by mitochondria. Data are the mean ± SEM (as this is the convention in the electron microscopy field) (^∗^*P* = 0.0186, *t*-test).

**Figure 4:** AQP4 overexpression improves neurobehavioral dysfunction in SAH mice. AAV-specific overexpression of AQP4 is beneficial to the early recovery of neurological function after SAH. (a) Garcia neuroscore. *n* = 12 per group (ANOVA *F*(15,220) = 16.37*P* < 0.0001; ^∗^*P* = 0.0296, post hoc Tukey's test). (b, c) Foot fault test of the left forelimb and left hind limb. *n* = 12 per group (ANOVA *F*(15,220) = 28.88*P* < 0.0001; ^∗∗^*P* = 0.0079, ^∗^*P* = 0.0133, ^∗∗∗^*P* < 0.001; post hoc Tukey's test. ANOVA *F*(15,220) = 29.60*P* < 0.0001; ^∗∗∗^*P* ≤ 0.001, ^∗^*P* = 0.0207, ^∗∗^*P* = 0.0038; post hoc Tukey's test). (d, e) Adhesive removal test. *n* = 12 per group (ANOVA *F*(15,220) = 28.24*P* < 0.0001; ^∗∗^*P* = 0.0066, ^∗∗^*P* = 0.0019, ^∗∗∗^*P* < 0.001; post hoc Tukey's test. ANOVA *F*(15,220) = 21.80*P* < 0.0001; ^∗^*P* = 0.0174, ^∗∗^*P* = 0.002, ^∗^*P* = 0.0154, ^∗∗∗^*P* < 0.001, post hoc Tukey's test). (f) Rotarod test. *n* = 12 per group (ANOVA *F*(15,220) = 188.2*P* < 0.0001; ^∗∗∗^*P* < 0.001, ^∗^*P* = 0.0197; post hoc Tukey's test). Data are the mean ± SD, SAH+AAV-AQP4 group vs. SAH+vector group.

**Figure 5:** Neurobehavioral ability was negatively correlated with transferrin brain content in SAH mice. Correlation analysis between the expression of transferrin in brain tissue and behavior at 24 hours after SAH. (a) Correlation analysis between the expression of transferrin in brain tissue and the modified Garcia neuroscore 24 hours after SAH. *n* = 6 per group. (b, c) Correlation analysis between the expression of transferrin in brain tissue and the stomping rate of the contralateral forelimb and hindlimb 24 hours after SAH. *n* = 6 per group. (d, e) Correlation analysis between the expression of transferrin in brain tissue and the time of sticker touch and avulsion 24 h after SAH. *n* = 6 per group. (f) Correlation analysis between the expression of transferrin in brain tissue and the stick time 24 h after SAH. *n* = 6 per group.

**Figure 6:** The mechanism of AQP4 involvement in early brain injury after SAH. In the early stage of SAH, transient disturbance of microcirculation and transferrin induced neuronal oxidative stress and iron uptake, leading to neuronal ferroptosis. Overexpression of AQP4 can improve SAH-induced AQP4 depolarization and transferrin infiltration and thus improve neuronal ferroptosis and neurological dysfunction.

## Data Availability

The data presented in this study are available on request from the corresponding author.

## Abbreviations

AQP4: Aquaporin 4
EBI: Early brain injury
PVS: Perivascular space
SAH: Subarachnoid hemorrhage.

## Supplementary Materials

Supplementary 1 Table S1: total mortality and exclusion rates of experimental mice. Table S2: detailed AQP4 overexpression adenoassociated virus information. Table S3, S4, and S5; resource identifiers for antibodies. Figure S1: qPCR revealed that AQP4 mRNA expression in AAV-APQ4 group was higher compared with the vector group. The expression level of AQP4-mRNA (NM_009700.3) after AAV-AQP4 treatment was detected by qPCR analyses. *n* = 6 per group. Data are the mean ± standard deviation (SD) (*t*-test *t* = 2.320, ^∗^*P* = 0.0427). Figure S2: schematic diagram of whole brain pictures and sampling sites of sham group and SAH group. The brain tissues were collected from the base of the temporal lobe and stored immediately −80°C for Western blot. Coronal brain sections containing the basal temporal lobe were used for PI staining.

Supplementary 2 Full western blot lane.
